RETRACTED

# Network Information Security Platform Based on Artificial Intelligence for the Elderly's Health “Integration of Physical, Medical, and Nursing Care”

**DOI:** 10.1155/2022/5975054

**Published:** 2022-05-27

**Authors:** Zongyou Yang, Siyong Xia, Sheng Feng

**Affiliations:** ^1^Department of Physical Education, Chongqing Jiaotong University, Nanan, 400074 Chongqing, China; ^2^School of Physical Education, Southwest University, Beibei, 400700 Chongqing, China; ^3^Physical Education Department of Chongqing Medical and Pharmaceutical College, Chongqing 401331, China

## Abstract

With the development of my country's economy and society and the improvement of civilization, the silver wave has gradually come. The country has launched a multifaceted pension model, such as institutional pension, home-based pension, and pension real estate. With the increasing aging of the population, traditional elderly care services can no longer meet the growing needs of the elderly. This research mainly discusses the construction of a network information security platform based on artificial intelligence for the elderly's health “integration of physical, medical, and nursing care.” The platform consists of five modules: health records, follow-up plans, remote training, health education, and remote consultation. Each module is equipped with a corresponding main interface and/or subinterface. Some modules also have submodules as needed. The structure is reasonable, and the interface is displayed. The combined medical care service model is divided into medical care, care care, and medical care. Among them, the medical care model mainly provides long-term comprehensive care services for the disabled, demented, semidisabled, and other elderly groups. The support-oriented model is mainly for self-care or semi-self-care elderly groups, providing rehabilitation monitoring and life care services. In terms of the overall effect of the platform, 13 users (81.25%) gave a high evaluation of the overall effect of the platform. This research will promote the development of the smart elderly care industry.

## 1. Introduction

In order to alleviate the problems caused by an aging society, my country has invested in the establishment of a series of elderly apartments, but because it is in its infancy, there are still many areas that need to be improved, especially in terms of demand that are limited to regular meals and housing. And so on, the requirements for the elderly's physical condition monitoring, behavioral status monitoring, and medical recovery have not been well realized.

With the increasing degree of aging in my country, old-age care has become a series of serious problems brought about by the aging process in China. On the premise of ensuring the health of the elderly, it combines intelligent technology to improve the living environment and lifestyle of the elderly, thereby improving living standards of the elderly. The research on the medical and nursing integrated network information security platform can meet the abovementioned innovative functions and guarantee functions, which has very important research significance.

RETRACTED

Information technology, artificial intelligence, and Internet technology were applied to the elderly care service industry, informatization of elderly care services, innovation and integration of elderly care service institutions at all levels, upgrading of traditional elderly care service industries, and improvement of service quality and diversity. Artificial intelligence technology affects all aspects of us. Makridakis believes that industry and the digital (information) revolution have had a significant impact on almost all aspects of society, life, companies, and employment. He will be able to use the Internet to buy goods and obtain services from anywhere in the world and take advantage of the unlimited additional benefits of the widespread use of artificial intelligence inventions. Although his research avoids the dangers and disadvantages of increased unemployment and increased wealth inequality, it cannot guarantee that it will provide huge opportunities for new products/services and huge increases in productivity [1]. Liu et al. believe that Fuzzy Petri Net (FPN) is a potential modeling technique for knowledge representation and reasoning in rule-based expert systems. In view of this constantly evolving research field, their work provides an overview of improved FPN theories and models from the perspectives of reasoning algorithms, knowledge representation, and FPN models. In addition, they also investigated the application of FPN in solving practical problems in various fields. Although they provided insights and a robust roadmap for further research in this field, the research still lacks innovation [2]. Etminaniesfahani et al. introduce a new metaheuristic algorithm. The Fibonacci indicator algorithm proposed by them has been verified on multiple benchmark functions of up to 100 dimensions, and it can converge and search with algorithms such as DE extension, PSO extension, ABC, ABC-PS, CS, MCS, and GSA. Comparing global optimal capabilities in different research fields, they finally demonstrated the performance of the algorithm through two engineering design problems. Although the application of their proposed Fibonacci indicator algorithm in a wide range of benchmark functions shows its ability to deal with difficult optimization problems, the algorithm is not very smart [3]. Kupcsik et al. believe that in robotics, low-level controllers are usually used to allow robots to solve specific tasks in a fixed environment. In order to adapt the strategy to the new context, they use the hierarchical approach by learning the upper-level strategy that generalizes the low-level controller to the new context. They proposed a new model-based context strategy search algorithm, which can generalize low-level controllers and is data-efficient. Although the learning framework they proposed accelerates the learning process by two orders of magnitude, while learning high-quality strategies, the research process is too complicated [4]. The state has issued a series of documents and policies, pointing out that it is necessary to promote the connection between medical and health care and elderly care service models and to explore new models of elderly care services.

RETRACTED

In today's social context, the problem of old-age care is becoming more and more prominent. With the support of pension policies in recent years, pension institutions have emerged, and more and more elderly people have favored and chosen pension institutions. The platform consists of five modules: health records, follow-up plans, remote training, health education, and remote consultation. Each module is equipped with a corresponding main interface and/or subinterface. Some modules also have submodules as needed. The structure is reasonable, and the interface is displayed, which is friendly and has stable operation of the system and convenient and quick operation. The user enters the platform by entering the user name and password granted and uses each module of the platform to realize the creation, editing, query, and viewing of health files; the creation, editing, query, and viewing of follow-up plans; remote training-related videos, courseware, and examination questions uploading, viewing, and downloading online; and uploading, viewing, and downloading health education-related documents, remote consultation application, review, and query functions. It is suggested to innovate the development model of the old-age service industry based on the national conditions, with the government as the leading role, the market to participate, and the development of basic old-age services as the core. At the same time, actively publicize, mobilize all social forces to join, and raise funds.

## 2. Research Method

### 2.1. Artificial Intelligence

Driven by smart technology, in the process of continuous development, some regions continue to integrate the latest smart technologies such as big data, artificial intelligence, and deep learning and reasonably add them to the original system, which is in depth with home care, community care, and institutional care, integrating, exploring, and developing a variety of hobbies and convenient services that can satisfy the elderly and even the elderly living alone and gradually form a new elderly care service system under smart elderly care, so that elderly care services can benefit more elderly people and promote the service line combination of online and offline, software and hardware, information and service, and technology and personnel. “Smart elderly care” can monitor the health of the elderly in an all-around way. For example, wrist sphygmomanometers, watch-type GPS locators, etc., can not only monitor the physical condition of the elderly anytime, anywhere, but also know their activity trajectories.

RETRACTED

The evaluation of the effect of information interaction in the context of smart medical care is not only a measure to measure the state of user information exchange and interaction but also the direction of the development strategy of smart medical care. It can be an in-depth analysis of the essential needs of their own information interaction in the context of smart medical care and their important impact on the future development of medical care. At the same time, the evaluation of the effect of information interaction in the context of smart medical treatment can guide smart medical platforms and institutions to enhance their core competitiveness, provide high-quality services, and promote the dynamic adaptation and organic integration of smart medical platforms and institutions, users, and the smart medical context. It goes without saying.

By integrating and optimizing medical resources and pension resources, establishing a collaborative and innovative comprehensive service platform, and exploring a sound “integration of medical care and nursing care” service model and effective long-term care methods, we can provide a reference for the public health service topic of smart elderly care. The evaluation system of information interaction in the context of smart medical treatment runs through the entire medical process. It should be a complete scientific system, including the comprehensiveness of the user subject, as well as the integrity and systemicity of information interaction. The results of the effect evaluation should be able to reveal the roles and connections between various levels, various dimensions, and various indicators. These indicators are effective for users, and their internal connections can be fully presented through some form of association. The evaluation process and results also need to maintain integrity and reveal user information interaction through hierarchical and structured result presentation, so that the results can maintain objectivity and authenticity. Normalize each column of the judgment matrix, namely [5],

(1) $$\begin{array}{c} b_{mn}=\frac{a_{mn}}{\sum_{i=1}^{n}a_{mn}}\;\left(m,n=1,2,3,\cdots ,n\right). \end{array}$$

After normalization, the sum of the elements in each column is 1. The normalized judgment matrix of each column is added by row, namely [6],

(2) $$\begin{array}{c} V=\overset{N}{\underset{J=1}{\sum }}B_{mn}\;\left(m,n=1,2,3,\cdots ,n\right). \end{array}$$

The intelligent elderly care system is based on the Internet of Things technology, and electronic chip devices are implanted in the home elderly care equipment, so that the daily life of the elderly is in a remote monitoring state. Normalize the vector *V* = [*v*_1_, *v*_2_, ⋯,*v*_*n*_]^*T*^ [7]:

(3) $$\begin{array}{c} w_{i}=\frac{v_{i}}{\sum_{i=1}^{n}v_{i}}\;\left(i,j=1,2,3,\cdots ,n\right). \end{array}$$

Calculate the largest characteristic root *λ*_max_ of the judgment matrix. Calculate the consistency index CI [8]:

(4) $$\begin{array}{c} \text{CI}=\frac{\lambda -n}{n-1}. \end{array}$$

Calculate the consistency ratio CR [9]:

(5) $$\begin{array}{c} \text{CR}=\frac{\text{CI}}{\text{RI}}. \end{array}$$

To optimize the effect of information interaction from the user's perspective, it is necessary to take the actual needs of users as the starting point and guide users to actively participate in smart medical information interaction activities. On the one hand, it is necessary to clarify the needs and expectations of users to participate in smart medical care, so as to ensure the enthusiasm and initiative of users to participate in smart medical information interaction activities; on the other hand, it is necessary to improve user information literacy to ensure that users can perform in the context of smart medical care. Interactive behavior of high-quality medical information [10]:

(6) $$\begin{array}{c} S\left(p\right)=\exp\left(-\frac{{\left\|p-X\right\|}_{2}^{2}}{\sigma^{2}}\right), \end{array}$$

(7) $$\begin{array}{c} S\left(p\right)=\max S^{*}\left(P\right). \end{array}$$

*P* is the amount of information, and *S*(*p*) is the entropy of information exchange [11].

RETRACTED

### 2.2. Combination of Medical and Nursing Care

Closely combine the basic life care and medical and health services of the elderly, so that they can enjoy convenient and high-quality medical and health care services in the process of providing for the elderly, that is, treatment when they are ill and convalescence when they are free, so as to improve the quality of life of the elderly. The old-age care model of the combination of medical and elderly care can connect elderly care institutions, society, communities, and families together and provide diversified elderly care services for the elderly. The services include life care, entertainment, health care, and long-term care. Its purpose is to provide diversified elderly care services for all types of elderly.

The elderly can enjoy elderly care services in various relevant places. The medical care integration model can better provide the elderly with advanced medical technology, equipment, and professional medical personnel, bring better and richer elderly care services to the elderly, and improve the quality of their elderly life. The old-age service model of the combination of medical and elderly care is aimed not only at the elderly who are suffering from diseases but also for the elderly who can take care of themselves; they can get satisfaction from the old-age services and the prevention and control of diseases. Elderly people suffering from illnesses can get better recovery and control through this old-age care service model that combines medical and elderly care.

There are many different classification standards for the medical and elderly care service model. According to the different positioning of “medicine” and “nourishment,” the combined medical care service model can be divided into medical care, care care, and medical care. Among them, the medical care model is mainly for disability and dementia. Elderly groups such as semidisabled need to provide long-term comprehensive care services, which are common in traditional medical institutions; the support-based model is mainly for self-care or semi-self-care elderly groups, which need to provide rehabilitation monitoring and life care services, which are common in nursing homes or community welfare homes, etc.; the mode of equal emphasis on medical care and care is mainly for self-care, just-needed care, and all-stage elderly groups, which need to provide services such as health care and life care, which are commonly found in new independent elderly communities or nursing apartments. The medical care integration model is shown in Figure 1.

Using *A* as the criterion-level judgment matrix, normalize each column of *A* to [12]

(8) $$\begin{array}{c} W_{ih}=\frac{a_{ih}}{\sum_{j=1}^{h}a_{ih}}. \end{array}$$

Sum up *W*_*ih*_ according to the line to get [13]

(9) $$\begin{array}{c} W_{i}=\overset{n}{\underset{j=1}{\sum }}W_{i}. \end{array}$$

Normalize *W*_*i*_ [14]:

(10) $$\begin{array}{c} \lambda =\frac{1}{n}\overset{n}{\underset{i=1}{\sum }}\frac{{\left(bw\right)}_{i}}{w}. \end{array}$$

Here, in order to judge the effectiveness of CI, we define a concept called random consistency RI, which is used to help researchers have a limit on CI [15]:

(11) $$\begin{array}{c} \text{RI}=\frac{{\text{CI}}_{1}+{\text{CI}}_{2}+\cdots +{\text{CI}}_{N}}{n}. \end{array}$$

The realization of artificial intelligence empowered community home care services depends on the development of artificial intelligence technology. The artificial intelligence community needs to strengthen the collection capabilities of elderly care data and improve the storage and computing capabilities of the elderly care information platform. At the same time, the intelligence of the pension algorithm model must be improved. It is necessary to not only improve the instrumental characteristics of AI-enabled community home care services but also reflect the humanized characteristics of artificial intelligence-enabled community home care services. The sample is represented as points distributed on the three-dimensional space *S* [16]:

(12) $$\begin{array}{c} \left(\phi_{ol}^{1},\phi_{om}^{1},\phi_{on}^{1}\right),\left(\phi_{ol}^{2},\phi_{om}^{2},\phi_{on}^{2}\right),\cdots ,\left(\phi_{ol}^{n},\phi_{om}^{n},\phi_{on}^{n}\right). \end{array}$$

Define the two-dimensional properties of Gaussian kernel local density and distance for the point, which are, respectively, denoted as [17]

(13) $$\begin{array}{c} \vartheta =\underset{jI\left\{S\right\}}{\sum }e^{-\left(d_{ij}/d\right)2},\;d_{c}>0. \end{array}$$

The total number is *N* = *τ*(*τ* − 1)/2, in ascending order [18]:

(14) $$\begin{array}{c} N=\frac{\tau \left(\tau -1\right)}{2}. \end{array}$$

RETRACTED

### 2.3. Construction of an Integrated Network Information Security Platform for Medical and Nursing Care

The platform is composed of five modules: health records, follow-up plan, remote training, health education, and remote consultation. Each module has a corresponding main interface and/or subinterface. Some modules also have submodules as needed. The structure is reasonable, and the interface is displayed and has a friendly and stable operation of the system and convenient and quick operation. The user enters the platform by entering the user name and password granted and uses the various modules of the platform to realize the creation, editing, query, and viewing of health files; the creation, editing, query, and viewing of follow-up plans; remote training-related videos, courseware, and examination questions upload, online viewing, and downloading; uploading, online viewing, and downloading of health education-related documents; and remote consultation application, review, and query functions. The platform login interface is shown in Figure 2.

1. *Health File Module*. The health file module displays the main interface by default and displays the health files of the elderly in the form of a list, which is simple and clear at a glance. Through list reading, you can quickly get the key information of a certain health file, such as file number, name, age, file establishment time, and chronic disease status; through the ascending and descending order next to the key information, you can sort the key information, such as sorting by age from big to small, quickly understand the information of the oldest elders, and grasp the age distribution range of the elders in the community. The health file list has a query function, which can be classified and searched according to conditions such as gender, chronic disease, and file establishment time and can also be searched according to file number, name, and ID number and can also be comprehensively searched for multiple conditions. The comprehensive use of functions facilitates community medical staff to quickly obtain key information about the elderly and to understand the health status of the elderly in time. Different color signs of different types of elderly are prominent and clearly displayed, which is convenient for quickly obtaining the classification level of the elderly and also avoids the monotony of the interface and relieves visual fatigue. There are 5 subinterfaces under the main interface, which are basic personal information, health examination, mental state, depression state, and self-care ability. Through the filling and viewing of each subinterface, the establishment and view of the elderly health files are completed. The combined use of drop-down menus and option buttons in the subinterface reduces the frequency of keyboard use, saves information filling time, improves information accuracy and work efficiency, and is particularly important for the insufficient allocation of medical staff in community hospitals. The option setting of the evaluation form entry assigns points. When the entry information is filled in, the system automatically generates the evaluation total score and evaluation level, reducing the process of manual score calculation, improving the efficiency and accuracy of the evaluation, and making the nursing management work more scientific, standardized, and efficient.
2. *Follow-Up Plan Module*. This module contains 3 submodules, namely, hypertension follow-up plan, diabetes follow-up plan, and special elderly follow-up plan; each submodule contains 1 main interface and 3 subinterfaces, which are follow-up records, follow-up information, and follow-up rules. The researcher adopted a similar design for each submodule, only the display content is different, and the same is true for each interface. This design makes the form of the module and interface more unified, clear, and simple and easy to operate; it also avoids the difficulty and cumbersome nursing management work caused by the module or interface being too complicated, which affects the effect of the platform. The main interface displays follow-up plans in the form of a list. Only the name, age, follow-up type, number of follow-ups, next follow-up time, and other important information of each follow-up plan are displayed in the list, which is simple and clear and easy to read quickly. The paging display of the follow-up plan bar not only improves the loading speed of the page, reduces the opening time of the page, and increases the timeliness of the user's visit but also avoids the bad experience brought to the user by the information listing, makes the important information prominent, and improves the browsing experience convenience. Click on a follow-up plan to view all follow-up records of someone. The follow-up records are also displayed in the form of a list. Click on a follow-up record to view the detailed information of a certain follow-up of someone. Click the “rules” button to enable the follower to quickly understand the corresponding chronic disease follow-up plan, each follow-up subtype, and its corresponding follow-up cycle, provide a reference for the follower, ensure the correct formulation of the follow-up cycle for the elderly, and achieve the health of the elderly real-time observation and dynamic tracking of the situation.
3. *Remote Training Module*. The remote training module contains a main interface and 3 subinterfaces. The conversion between the main interface and the subinterfaces is realized by clicking on the corresponding fields. The nodes of the main and subinterfaces are distinct, and the conversion is smooth to ensure that the information is clear. The details are appropriate, and it is convenient for users to browse and obtain the best information according to their needs. The training theme of the main interface includes the training sequence, which clearly shows the current training sequence and the total number of remote trainings. By viewing the video subinterface, courseware subinterface, and test question subinterface, you can obtain AVI videos, PPT courseware, and word test questions of related training topics in turn. Not only can you watch online, but also you can “download and print” through the upper right corner of the subinterface button to download and print the corresponding materials, which is convenient for community nurses to study at flexible times and different occasions, reasonable arrangement of study plans, and improvement of the efficiency and enthusiasm of distance training.
4. *Health Education Module*. The health education module includes the main interface and a subinterface. The main interface displays health education information in the form of a list, including sequence and title, so that community nurses can obtain corresponding health education materials according to their needs. Each health education material contains comprehensive knowledge of definition, etiology, classification, symptoms, treatment, and nursing. Community nurses strengthen their comprehensive understanding of the disease through the study of health education materials, thereby improving their own health education ability and level. Through the “download” and “print” buttons, the corresponding health education materials can also be downloaded and printed, which is convenient for community nurses to store safely and learn flexibly.
5. *Remote Consultation Module*. The remote consultation module contains 3 submodules, which in turn are consultation application, consultation review, and consultation view. Community nurses use the keyboard or drop-down list to enter the complete information in three parts: basic patient information, patient condition introduction, and consultation purpose, and complete the consultation application initiated at our hospital. The setting of the drop-down list reduces the number of keyboard input and saves the time for filling out the consultation application, which not only improves the work efficiency but also ensures the accuracy of the consultation application information. Consultation experts can query, view, and fill in the corresponding consultation review results on the consultation review interface, while community nurses cannot operate on the consultation review interface; community nurses can query and view the review status and review of the consultation application that has been initiated through the consultation review interface. For the result, the setting of different user access permissions on the consultation review interface ensures the standardized management and safety of the system, which not only ensures the security and authenticity of the data but also protects the privacy of the hospital and patients [19]. The constructed platform architecture is shown in Figure 3.

RETRACTED

## 3. Results

In this part of the study, a total of 420 questionnaires were distributed, and 410 valid questionnaires were recovered, with an effective recovery rate of 97.62%. Among the 410 community elders, there were 166 males (40.49%) and 244 females (59.51%); 189 cases (46.10%) aged 60-69, 150 cases (36.59%) aged 70-79, and 71 cases (17.32%) aged 80 and older; 133 were healthy cases (32.44%), and 277 were sick cases (67.56%), of which 55.96% of the elderly suffer from two or more diseases at the same time, and the top three chronic diseases are hypertension (35.40%), diabetes (21.50%), and coronary atherosclerotic heart disease (19.00%). The general information about the elderly in the community is shown in Table 1.

The total score of community elderly care needs for home care is 60.24 ± 11.16 points, showing a relatively high level; the total scores of each dimension are disease care 25.90 ± 7.00 points, disease prevention 11.95 ± 1.74 points, and health promotion 22.39 ± 4.35 points. The average score of each dimension shows that disease prevention needs have the highest score, followed by health promotion needs, and disease care needs have the lowest score.  Table 2 shows the scores of home care needs for the elderly in the community.

Combine those who selected “not needed,” “not much needed,” and “indifferent” in the questionnaire and record them as no need for the nursing service item; combine those who selected “need” and “very in need” and record them as correct There is a demand for this nursing service item.  Table 3 shows the ranking of demand for home care services for the elderly in the community.

A single factor analysis of the home care needs of the elderly in the community with different demographic characteristics found that the older the age, the higher the demand; the higher the education level, the higher the demand; married elderly people have higher demand than unmarried, divorced, and widowed elderly; for income and expenditure, demand for the surplus is higher; the demand of the sick elderly is higher; the self-care ability is negatively correlated with the demand; the lower the self-care ability, the higher the demand. The single factor analysis of the demand for home care for the elderly in the community is shown in Table 4.

The factors influencing the needs for home care for the elderly in the community are disease, age, income and expenditure, education, marital status, and self-care ability according to the standard regression coefficient. The multiple linear regression analysis of the demand for home care for the elderly in the community is shown in Table 5.

There were 28 males and 60 females in the test group, with an average age of 73.56 ± 6.30 years, and 38 males and 54 females in the control group, with an average age of 73.74 ± 6.04 years. The comparison of the general data of the two groups of community elderly at baseline was not statistically significant (*P* > 0.05), indicating that the general data of the two groups of community elderly at baseline were comparable. The situation of the elderly in the two groups of communities is shown in Figure 4.

RETRACTED

*Effectiveness evaluation*: in terms of operating convenience, 13 (81.25%) users thought that the platform was friendly and easy to operate; in terms of system stability, 4 (25.00%) users encountered network instability, freezes, and lags during use and black screen and other situations; in terms of application value, 14 (87.50%) users believe that through this platform, they can learn advanced nursing technology and experience in general hospitals, provide more high-quality and efficient nursing services for the elderly, and can also deal with problems that the institution cannot solve in a timely manner. In terms of the overall effect of the platform, 13 users (81.25%) have a high evaluation of the overall effect of the platform. Another 3 users made suggestions to the platform. The content includes that the follow-up time is more individualized and not easy to remember in time. It is recommended that when the follow-up date is approaching, the system pops up a prompt message; when the health file information is completed and submitted, the system does not display the submission status; it is recommended to add the submission status prompt box; and increase the statistical function of the query results. The evaluation results of the platform are shown in Figure 5.

One month later, the differences in the total scores of the health self-management ability of the two groups of community elders and the scores of each dimension were statistically significant (*P* < 0.05). After one month of intervention, the experimental group had better health self-management ability than the control group. The result after 1 month is shown in Figure 6.

After the intervention for 3 months, the difference in satisfaction of the two groups of community elderly home care services in all aspects was statistically significant (*P* < 0.05). After the intervention for 3 months, the test group's satisfaction with home care services was higher than that of the control group. The intervention satisfaction after 3 months is shown in Figure 7.

After 6 months of intervention, the difference in satisfaction between the two groups of community elderly home care services in all aspects was statistically significant (*P* < 0.05). After 6 months of intervention, the test group's satisfaction with home care services was higher than that of the control group. Intervention 6 results after one month are shown in Table 6.

## 4. Discussion

In reality, the status quo in most areas is still the separation of medical care and support and their own governance. Even if the medical care integration model is established, the development effect is not very satisfactory. As a result, the elderly cannot truly enjoy their old age, whether it is physical or not physical. Mental health should be actively dealt with, which shows that the medical care integration model can well solve the problem of the health needs of the elderly, which also confirms the necessity of the construction of the medical care integration model. Even if the abovementioned series of problems are solved, the constructed medical care integration service model may still have problems such as resource imbalance, waste of resources, and low utilization efficiency. How to use the concepts and theories of artificial intelligence to be organic with the medical care integration service model combined and the real realization of artificial intelligence in the elderly care service system is also a question worth pondering [20, 21].

RETRACTED

Medical care integration services can be seen as a commodity or a quasipublic product. Therefore, specific to the provider, the provider can be a for-profit organization or a nonprofit organization, or it can be a public sector such as the government. In the process, it is clear that it is not enough to rely solely on a certain aspect of the force. As a service with a more prominent quasipublic product attribute, it must be led by the government, and the effective forces and resources of all aspects must be integrated. It requires the government, profit, and nonprofit organizations to work together to meet the growing demand for services. In terms of service targets, the medical care integration service should not be aimed at all aging people. It should be said that the medical care integration service is essentially an organic system with two levels. The first is “medical.” At the level, the medical treatment here involves all aspects, and more is for the aging groups who suffer from chronic diseases and need long-term real-time monitoring; the “nourishing” level is mainly for the daily life of the aging people and should also be taken care of and contains its spiritual needs and psychological needs. Therefore, the target of medical care integration service should be a group with high demand for medical services and certain obstacles to living ability. Only by accurately positioning the service target can we use resources better and more efficiently. The service content should not be based on the traditional daily life care of the aging population. In addition to meeting the physical needs of the aging population, it should pay more attention to the psychological and spiritual needs of the population. In the interpretation of connotation, not only the physical integrity but also the psychological and social adaptability are more important [22]. In addition, medical services should not be separated from the old-age service system but should be integrated into it, and even for specific groups of people, medical services should be the mainstay, and medical services should be regarded as one of the equally important service contents [23, 24].

RETRACTED

Based on the analysis of the different levels of the artificial intelligence medical care integration service model, it should also be analyzed in combination with the actual situation in my country. The characteristics of my country's urban and rural areas are very obvious, and the differences are significant. The urban elderly population is relatively better than the rural elderly in all aspects. The population and the educational level of the urban elderly population are generally higher than that of the rural elderly population; these are all factors to be considered [25]. In addition, in the precise segmentation of service targets, we should consider that the current needs of the elderly group are actually multilayered and diverse. Not all elderly groups have “nourishing” service needs, which are completely relevant to life. Or for groups who are basically able to take care of themselves, more needs are the needs for “medicine”; even if it is the need for “medicine,” it is only for the elderly who are diagnosed or self-reported with chronic diseases, and there is medical integration. The service needs are often disabled or partially disabled elderly people and elderly people with or without chronic diseases. These should be carefully divided and considered when constructing the artificial intelligence medical care integration service model. The differences are different. The population adopts different service systems and models, which is the integration of artificial intelligence medical care in a complete sense [26–29].

## 5. Conclusion

This article takes the perspective of artificial intelligence as the starting point, first analyzes the current situation of China's elderly care service demand and supply, and points out that China's current population aging status and future development trends are not optimistic, and it is for the improvement and further development of China's elderly care service system. Put forward an unprecedentedly huge challenge and at the same time analyze in detail several needs of the elderly themselves, mainly including economic needs, health and medical needs, life care needs, and mental and psychological needs; from the number of elderly care service institutions and related elderly care services, the policy is combed to have a more comprehensive understanding of the current status of the supply of elderly care services, and at the same time, it briefly introduces the development history of China's elderly care service system, etc., and discusses the construction of artificial intelligence+medical care based on a series of issues such as the contradiction between demand and supply. The necessity of the integrated service model, starting with the traditional medical care integrated service model case and public perception, analyzes the operating mode of the medical care integrated service organization and on this basis analyzes its advantages, disadvantages, opportunities, and challenges. The traditional medical care integrated service model has many drawbacks, and it cannot fundamentally meet the diversified needs of the elderly, and it also brings certain pressure to the society. Based on this, it has triggered the exploration of the artificial intelligence+medical care integrated service model.

RETRACTED

## Figures and Tables

**Figure 1:** Medical care integration model.

**Figure 2:** Platform login interface.

**Figure 3:** Platform construction architecture.

**Figure 4:** The situation of the two groups of elderly in the community.

**Figure 5:** Evaluation results of the platform.

**Figure 6:** Results after 1 month of intervention.

**Figure 7:** Satisfaction after 3 months of intervention.

**Table 1:** General information on the elderly in the community.

Parameter	Project	Number of cases	Composition ratio (%)
Income and expenditure	Have balance	78	19.02
	Break even	275	67.07
	Make ends meet	57	13.90
Medical insurance type	Own expense	37	9.02
	Rural health insurance	271	66.10
	Urban medical insurance	81	19.76
Illness	Business insurance	133	5.12
	Health	277	32.44
	Sick	78	67.56

**Table 2:** The scores of home care needs of the elderly in the community.

Project	Overall demand	Illness care	Prevent disease	Health promotion
Total score	60.24 ± 11.16	25.90 ± 7.00	11.95 ± 1.74	22.39 ± 4.35
Average score	3.54 ± 0.66	3.24 ± 0.88	3.98 ± 0.58	3.73 ± 0.72

**Table 3:** Ranking of demand for home care services for the elderly in the community.

Parameter	Number of cases in demand	Percentage (%)	Rank
Income and expenditure	366	89.27	1
Medical insurance type	352	85.85	2
Illness	33 1	80.73	4
Own expense	330	80.49	5
Rural health insurance	315	76.83	6
Urban medical insurance	31 2	76.10	7
Business insurance	302	73.66	8
Health	292	71.22	9
Sick	280	68.29	10

**Table 4:** Single factor analysis of the demand for home care for the elderly in the community.

Project	Number of cases	Mean ± standard deviation
Local	331	60.34 ± 11.17
Out of town	79	59.82 ± 11.20
Elementary school and below	110	57.55 ± 14.08
Junior high school	242	61.15 ± 10.20
High school and above	58	61.53 ± 7.45

RETRACTED

**Table 5:** Multiple linear regression analysis of community elderly care needs at home.

Variable	*B*	Beta	15.126
Constant	56.669	—	7.109
Illness	8.228	0.346	5.202
Age	3.554	0.237	-5.983
Income and expenditure	-4.981	-0.225	3.595
Education	2.712	0.153	-2. 921

**Table 6:** Results after 6 months of intervention.

Project		Satisfaction	General	Dissatisfied
Instrument appearance	Test group	60	26	2
	Control group	46	34	12
Professional knowledge	Test group	58	28	2
	Control group	42	38	6
Service attitude	Test group	57	25	16
	Control group	43	33	6

## Data Availability

No data were used to support this study.
